# Flavonoids modulate multidrug resistance through wnt signaling in P-glycoprotein overexpressing cell lines

**DOI:** 10.1186/s12885-018-5103-1

**Published:** 2018-11-26

**Authors:** S. Mohana, M. Ganesan, N. Rajendra Prasad, D. Ananthakrishnan, D. Velmurugan

**Affiliations:** 1 Department of Biochemistry and Biotechnology, Annamalai University, Annamalai Nagar, Tamil Nadu 608 002 India; 2 Bioinformatics Infrastructure Facility (BIF), University of Madras, Guindy Campus, Chennai, Tamil Nadu India; 3 CAS in Crystallography and Biophysics, University of Madras, Guindy Campus, Chennai, Tamil Nadu India

**Keywords:** Wnt/β-catenin signaling, Flavonoids, Molecular docking, P-glycoprotein, Multidrug resistance, GSK 3β

## Abstract

**Background:**

Wnt signaling has been linked with P-glycoprotein (P-gp) overexpression and which was mainly mediated by β-catenin nuclear translocation. Flavonoids have already been reported as modulators of the Wnt/β-catenin pathway and hence they may serve as promising agents in the reversal of P-gp mediated cancer multi drug resistance (MDR).

**Methods:**

In this study, we screened selected flavonoids against Wnt/β-catenin signaling molecules. The binding interaction of flavonoids (theaflavin, quercetin, rutin, epicatechin 3 gallate and tamarixetin) with GSK 3β was determined by molecular docking. Flavonoids on P-gp expression and the components of Wnt signaling in drug-resistant KBCH^R^8–5 cells were analyzed by western blotting and qRT-PCR. The MDR reversal potential of these selected flavonoids against P-gp mediated drug resistance was analyzed by cytotoxicity assay in KBCH^R^8–5 and MCF7/ADR cell lines. The chemosensitizing potential of flavonoids was further analyzed by observing cell cycle arrest in KBCH^R^8–5 cells.

**Results:**

In this study, we observed that the components of Wnt/β-catenin pathway such as Wnt and GSK 3β were activated in multidrug resistant KBCH^R^8–5 cell lines. All the flavonoids selected in this study significantly decreased the expression of Wnt and GSK 3β in KBCH^R^8–5 cells and subsequently modulates P-gp overexpression in this drug-resistant cell line. Further, we observed that these flavonoids considerably decreased the doxorubicin resistance in KBCH^R^8–5 and MCF7/ADR cell lines. The MDR reversal potential of flavonoids were found to be in the order of theaflavin > quercetin > rutin > epicatechin 3 gallate > tamarixetin. Moreover, we observed that flavonoids pretreatment significantly induced the doxorubicin-mediated arrest at the phase of G2/M. Further, the combinations of doxorubicin with flavonoids significantly modulate the expression of drug response genes in KBCH^R^8–5 cells.

**Conclusion:**

The present findings illustrate that the studied flavonoids significantly enhances doxorubicin-mediated cell death through modulating P-gp expression pattern by targeting Wnt/β-catenin signaling in drug-resistant KBCH^R^8–5 cells.

**Electronic supplementary material:**

The online version of this article (10.1186/s12885-018-5103-1) contains supplementary material, which is available to authorized users.

## Background

Multidrug resistance (MDR) is a mechanism through which several cancer subtypes exhibit resistance to anticancer drugs resulted in the chemotherapy failure [1]. This MDR phenomenon is mainly associated with overexpression of membrane-bound molecular “pumps” that dynamically efflux out structurally and functionally different anticancer drugs from the tumor cells. The P-glycoprotein (170 kDa), belongs to ATP-binding cassette transporters family (ABC), confer resistance to various chemotherapeutic drugs [2]. Thus, inhibition of its drug transport function or modulation of its expression in cancer cells will be a novel strategy to overcome cancer multidrug resistance.

Existing data illustrated that natural flavonoids possess significant modulatory effects on drug resistance in cancer [3]. Recently, we systematically screened flavonoids against P-gp drug efflux function using calcein-AM drug efflux system and further observed flavonoids such as quercetin and rutin reverse MDR several folds in KBCHR8–5 cell lines [4]. Shtil et al.*,* 1994 demonstrated modulation of P-gp overexpression at the molecular level to overcome MDR in cancer cells [5]. The activation of Wnt/β-catenin signaling molecules leads to overexpression of P-gp which contributed to clinical MDR [6]. In the canonical pathway, β-catenin is phosphorylated and activated by a set of proteins which includes GSK-3β, axin and APC. Stabilized cytoplasmic β-catenin translocates from the cytoplasm to the nucleus and activates T-cell factor (TCF) transcription factors then subsequently activates ABCB1 overexpression [7]. Therefore, downregulation of Wnt/GSK 3β/β-catenin pathway possibly will reduce the P-gp expression and induce chemosensitization in drug-resistant cells. The GSK 3β is an important factor of Wnt/β-catenin signaling and pharmacological inhibition or modulation of GSK 3β expression might reverse the MDR in drug-resistant cells.

Numerous reports illustrate that flavonoids could able to modulate the Wnt pathway thereby increases to their antitumor effect against cancer cells [8, 9]. Kitagawa et al., (2004) illustrated the reversal potential of flavonoids on the function of P-gp in KB-C2 cells using daunorubicin and rhodamine-123 [10]. Herein, we investigated the chemosensitizing efficacy of selected flavonoids like theaflavin, rutin,, quercetin, epicatechin 3-gallate and tamarixetin in colchicines-selected KBCH^R^8–5 cell lines through targeting Wnt/GSK 3β/β-catenin pathway. To determine whether these flavonoids modulate P-gp mediated MDR, we carried out cell-based assays, transcriptome analysis and Wnt proteins expression in the presence or absence of these flavonoids in KB 3–1 and colchicine-selected KBCH^R^8–5 cell lines.

## Methods

### Molecular docking

Induced-fit docking was carried out to predict theaflavin, quercetin, rutin, epicatechin 3 gallate and tamarixetin binding interaction in the GSK 3β using Glide and prime modules [11]. Ligprep 2.3 module (Schrodinger) was used for the preparation of theaflavin, quercetin, rutin, epicatechin 3 gallate and tamarixetin. The 3D GSK 3β (PDB: 5HLN) structure was obtained from the PDB (http://www.rcsb.org). The Schrodinger software was used for GSK 3β preparation as per the procedure described previously [12].

### Chemosensitizing effect of flavonoids by MTT assay

We have analyzed the chemosensitizing potential of flavonoids by MTT assay [13]. KB 3–1, KBCH^R^8–5, MCF-7 and MCF-7/ADR cells (1X10^4^ cells/ well) were initially seeded in 96 well plates and kept incubated for 24 h. Further, cells were preincubated with or without the different concentration of flavonoids (1–10 μM per well) for 2 h, consequently, various concentrations of doxorubicin were added into the designated wells for 72 h. Then, MTT solution (4 mg/ml) was added and incubated for 4 h. Further, 100 μL of DMSO was added and the absorbance of formazan solution was measured at 570 nm using a multimode reader (Tecan, Austria).

### Western blot analysis

We have done western blot analysis to find out flavonoids mediated alteration of protein expression in KBCH^R^8–5 cells. The KBCH^R^8–5 cells (5 × 10^6^ cells) were lysed using RIPA buffer. The protein concentration was estimated using nanodrop spectrophotometer (Thermo Scientific Inc.). Proteins were separated by 12% SDS-PAGE then blotted to nitrocellulose membrane. Then, the blotted membranes were treated with 5% BSA at for 1 h. The membranes were then kept incubated at 4 °C overnight with monoclonal antibodies for P-gp (1:1000), Wnt (1:1000), GSK 3β (1:1000) (Santa Cruz, USA). Then, the membrane was incubated for 1 h with the horseradish peroxidase conjugated secondary antibodies. Then, the protein expressions were detected using chemiluminence western blot detection kit (Biorad, USA).

### qRT-PCR analysis of LRP6, FZD1, APC and axin expression

The mRNA expression of LRP 6, Frizzled (FZD) 1, adenomatous polyposis coli (APC) and axin, in KBCH^R^8–5 cells was analyzed using real-time PCR. cDNA was synthesized using 100 ng total RNA by RT^2^ First strand kit. Complimentary DNA was amplified (20 μL) using SYBR green master mix and 0.5 μM of the specific primers. Real-time PCR was carried out on Eppendorf master cycler (Eppendorf, Thermocycler, USA). The gene expression levels were normalized to 18S mRNA expression in each sample. The mean cyclic threshold (Ct) of each gene expression was accounted to measure the relative gene expression by employing the formula 2^-ΔΔCt^.

### Cell cycle analysis

After treatment with flavonoids and/or doxorubicin cells (1X10^6^cells/well) were trypsinized and washed with PBS. Then, the treated cells were fixed using cold 70% ethanol and incubated for overnight at 4 °C. After a single wash with PBS, the cells were incubated using 50 pg/ml of propidium iodide and 0.1 mg/ml of RNaseA for 30 min. After that, cells were kept incubated for 30 min in dark. The DNA content in each phase of the cell cycle was then analyzed using a FACS (BD Aria III, BD Biosciences) [14].

### PCR array

The total RNA was isolated using RNAeasy kit (Qiagen, India). The relative mRNA expression (RQ) pattern of 9 genes involved in drug resistance, cell cycle, apoptosis, and Wnt/β-catenin pathway were investigated by PCR array by SYBR Green PCR master mix (Qiagen, qRT-PCR array) on Eppendorf realplex PCR instrument. The gene expression in fold changes was plotted as clustergram using PCR data analysis.sabiosciences.com/pcr/ arrayanalysis.php.

## Results and discussion

The P-glycoprotein (ABCB1/MDR1) serves as key regulators in the efflux of chemotherapeutic agents [15]. Several recent findings indicate the link between Wnt/β-catenin pathway and the ABC transporters overexpression [16, 17]. Previously, it has been reported that Wnt5A regulates ABCB1 expression pattern through the non-canonical PKA/β-catenin pathway in drug resistant cancer cells [18]. Flavonoids have been reported to inhibit ABCB1 transporters that contribute to the development of MDR [19]. In this study, we investigated the reversal of P-gp mediated MDR via targeting the Wnt/β-catenin pathway by selected dietary flavonoids which show chemosensitizing property in our preliminary studies [4]. In this study, induced-fit docking reveals that flavonoids inhibit GSK 3β directly by interacting to the ATP binding site of the protein. Among the flavonoids studied theaflavin effectively interact with Ligand Binding Domain (LBD) of GSK 3β (− 85.58 kcal/mol) (Fig. 1; Additional file 1: Figure S1 and Table S1). The binding interaction of theaflavin against GSK 3β was compared with its cocrystal 65C (6-[(2-{[4-(2, 4-dichlorophenyl) -5-(4-methyl-1H-imidazole-2-yl) pyrimidin-2-yl] amino} ethyl) amino] pyridine- 3-carbonitrile) and VAL-135 was found to be contributed in the common hydrogen-bond interactions. The ATP-competitive GSK 3β inhibitors bind with GSK 3β by hydrogen bonding to the carbonyl and amino groups of the valine 135 amino acid and also to the carbonyl oxygen of Asp133 within the hinge area of the ATP-binding pocket [20]. Shin et al. (2007) established a hydroxyl group at C_7_ of the benzimidazole to generate hydrogen bonds to the amino group of Val 135 and the carbonyl group of the Asp 133 residue [21]. Additionally, Coffman et al. (2011) developed several GSK-3β inhibitors and these compounds interacts within the GSK-3β ATP site. Similarly, in our study, we found flavanoids binds within the ATP site of GSK-3β particularly with the Val 135 and Asp 133 residues of the hinge region [22]. Sivaraman (2015) screened GSK 3β inhibitors against flavonoids which shows Val 135 to be the major active amino acid which is present in all the docked compounds [23]. Johnson et al., (2011) showed molecular docking of citrus flavonoids with GSK-3β and found that quercetin effectively inhibits GSK-3β activity [24]. Moreover, Iftikhar and Rashid (2014) showed a pharmacophore model of flavonoids to generate potent inhibitors for targeting Wnt signaling pathway [25]. Therefore, the present results suggest that the flavonoids could interact with GSK-3β backbone amino acids Asp133 and Val135. Our in vitro findings along with findings of other investigators trigger us to experimentally prove the role of dietary flavonoids on the role of flavonoids Wnt/GSK-3β pathway to overcome MDR in cancer.

**Fig. 1:** **a**) Pymol observation of ligand binding domain (LBD) of GSK 3β with theaflavin. **b**) Ligplot representation illustrates hydrophobic and hydrogen bondig of GSK 3β with theaflavin

We observed that the Wnt and GSK-3β were activated in the colchicine-selected KBCH^R^8–5 cell lines. Activation of the Wnt signaling elements might lead to the overexpression of membrane P-gp. We found that β-catenin translocation into the nucleus in drug resistant KBCH^R^8–5 cells. This substantiates the role of Wnt/β-catenin in ABCB1 overexpression in the KBCH^R^8–5 cells (Fig. 2; Additional file 1: Figure S2). In this present study, flavonoids also decreased the expression of Wnt and GSK 3β in KBCH^R^8–5 cells. Further, flavonoids treatment prevented the translocation of β-catenin to the nucleus in the drug-resistant cells. Thereby, flavonoids downregulate P-gp overexpression in KBCH^R^8–5 cells; this was noticed in a dose-dependent manner (Fig. 2). Similarly, Park and Choi reported that binding of Tcf complexes with specific DNA binding sites has been suppressed by flavonoids through diverse mechanisms in colorectal cancer [26]. It has been well established that the down-regulation of the canonical Wnt/GSK-3β/β-catenin pathway is known to downregulates the P-gp expression in various cancer subtypes [27–31]. Previously, it has been reported that quercetin binds with β-catenin thereby block binding interaction between β-catenin and TCF [32].

**Fig. 2:** **a** and **b**. Wnt, GSK 3β and β-catenin mRNA and protein expression pattern in KB3–1 and KBCH^R^8–5 cell lines. Protein (Western blot) and mRNA (qRT-PCR) expression status of Wnt, GSK 3β, LRP6, FZD1, APC and axin in KBCH^R^8–5 cells. (**c**) theaflavin, (**d**) quercetin, (**e**) rutin, (**f**) epicatechin 3 gallate (E3G) and (**g**) tamarixetin. The protein levels were quantified by LI-COR Image Studio tool. The data denote means ± SD from three experiments. The protein expressions were normalized to the β-actin expression level. Gene expression was normalized with 18S and depicts quantification of three independent experiments (means ± S.D). Symbols not sharing a common symbol vary significantly at *p* ≤ 0.05 (DMRT)

In this study, flavonoids prevent the translocation β-catenin, thereby downregulates P-gp expression in KBCH^R^8–5 cells. The phosphorylation-dependent degradation of β-catenin prevented nuclear translocation and binding on the mdr1 promoter which downregulates P-gp by temozolomide acting like a Wnt-pathway inhibitor [33]. Wnt/β-catenin acts as a potential target to overcome resistance in cholangiocarcinoma [6]. Further, the FZD1 silencing significantly downregulated cytoplasmic and nuclear β-catenin expression levels and down-regulates the expression of MDR1/P-gp, thereby restored sensitivity to chemotherapy drugs [34]. Flavonoids are reported to block different components of Wnt signaling thereby reverses MDR [35]. Previously, it was illustrated that quercetin could regulates wnt signaling by affecting their pathway components in colon cancer cells, SW480 cells, leukemia and lymphoma cells [36]. Isoquercitrin inhibits glioblastoma proliferation through Wnt/β-catenin pathway [37]. Recently, Chen et al., (2018) showed quercetin enhances the efficacy of chemotherapeutic drugs in ABCB1, ABCC1 and ABCC2-overexpressing cells by regulating the FZD7/β-catenin signaling [16].

The Wnt/β-catenin signaling has been found to be related to the overexpression of ABC transporters [38, 39]. The β-catenin was found to be released from the APC/axin complex which activates transcription of the mdr1 gene. We observed that overexpression of mRNA patterns of ABCB1 and Wnt/β-catenin pathway components such as LRP 6 and GSK 3β in KBCH^R^8–5 cells (Fig. 2; Additional file 1: Figure S3). Flavonoids pretreatment also augment doxorubicin-induced apoptosis in KBCH^R^8–5 cell lines. Doxorubicin mediate apoptotic cell death by modulating signaling elements [40]. Previous report state that flavonoids augment cell cycle arrest in distinct phases of cancer [41]. Flavonoids significantly downregulate the mRNA expression of CDK2, BCL-XL and upregulate p53, CDKN1A, BAX in KBCH^R^8–5 cells (Fig. 3). The MDR1 promoter has also been affected by p53 which affects endogenous MDR1 expression [41]. In this study, we found that the studied flavonoids sensitize doxorubicin and upregulate p53 expression which subsequently induces apoptotic events in drug-resistant cells. Moreover, we observed that flavonoids pretreatment significantly augment the doxorubicin-mediated arrest at the G2/M phase of the cell cycle (Fig. 4). Flavonoids significantly enhance doxorubicin efficacy in drug-resistant KBCH^R^8–5 cells. Hence, we stated that downregulation of ABCB1 and subsequent modulation of doxorubicin-mediated cell cycle arrest and apoptotic signaling may be the reason for the chemosensitizing property of the studied flavonoids in P-gp overexpressing oral carcinoma cell lines. Thus, flavonoids enhanced doxorubicin efficacy through Wnt/β-catenin signaling and subsequently downregulates ABCB1 expression thereby promotes doxorubicin-induced G2/M arrest and apoptosis in multidrug-resistant KBCH^R^8–5 cells.

**Fig. 3:** Theaflavin, quercetin, rutin, epicatechin 3 gallate (E3G) and tamarixetin and/or doxorubicin on MDR-linked gene expression pattern in KBCH^R^8–5 cells. The mRNA expression levels of 9 genes involved in drug resistance and Wnt/β-catenin signaling were detected using qPCR. Clustergram was constructed using the SA Biosciences online tool using three independent experiments

**Fig. 4:** Effect of flavonoids on doxorubicin-induced cell cycle arrest. Theaflavin, quercetin, rutin, epicatechin 3 gallate (E3G) and tamarixetin treatment potentiates G2/M arrest in doxorubicin-treated KBCH^R^8–5 cells. The cells were exposed to 7 μM of doxorubicin alone or in combination with 10 μM of theaflavin, rutin, epicatechin 3-gallate, quercetin and tamarixetin for 24 h. Different cell cycle phases were monitored by flow cytometer

The P-gp overexpressing KBCH^R^8–5 cells exhibit 175-fold drug resistance to doxorubicin, compared to KB 3–1 cell line (Fig. 5). We observed that flavonoids considerably decreased doxorubicin resistance in KBCH^R^8–5 cell line (Table 1). We performed cell-based cytotoxic assays in the MCF-7 and MCF-7/ADR cell lines in the presence or absence of flavonoids (Fig. 6). MCF-7/ADR cell lines exhibit 27 fold resistances to doxorubicin, when compared to the parental MCF-7 cell lines (Table 2). Flavanoids considerably decreased the doxorubicin resistance in MCF-7/ADR cells when compared to the control MCF-7 cell lines. It has been found that 10 μM of flavonoids significantly reverse the P-gp mediated MDR in KBCH^R^8–5 and MCF-7/ADR cells as compared to other lower concentrations. Further, the MDR reversal potential of flavonoids was in the order of theaflavin > quercetin > rutin > epicatechin 3-gallate > tamarixetin. Therefore, the studied flavonoids prevent the nuclear translocation β-catenin through interacting with GSK 3β and different components of Wnt signaling pathway thereby downregulates P-gp overexpression in drug resistant oral carcinoma KB cells (Fig. 7).

**Fig. 5:** Chemosensitizing effect of the selected flavonoids in drug-resistant KBCH^R^8–5 cell lines. Concentration dependent curves of doxorubicin with or without flavonoids (1, 5 and 10 μM) in parental KB 3–1 and KBCH^R^8–5 cell lines were constructed. The IC_50_ values of KBCH^R^8–5 cell lines were equaled with parental KB 3–1 cells (Table 1). Data with error bars show the mean ± S.E.M of four experiments, each done in triplicate

**Table 1:** The concentration of flavonoids necessary for 50% inhibition (IC_50_ values). Data of mean ± SEM are from four analytical experiments, each conducted in triplicate. bFR: fold-drug resistance was derived by dividing the IC_50_ concentration for doxorubicin of KB 3–1 and KBCH^R^8–5 cells in the absence/presence of flavonoids by IC_50_ value for doxorubicin of KB 3–1 cells

Compound	KB 3–1		KB Ch^R^ 8–5	
	IC_50_ ± SEM^α^ (μM)	FR^b^	IC_50_ ± SEM^α^ (μΜ)	FR^b^
Doxorubicin	0.04 ± 0.01	[1.0]	7 ± 0.20	[175.0]
+ 1 μM Theaflavine	0.03 ± 0.01	[0.8]	3 ± 0.04	[75.0]
+ 5 μM Theaflavine	0.02 ± 0.01	[0.5]	0.6 ± 0. 03	[15.0]
+ 10 μM Theaflavine	0.02 ± 0.01	[0.5]	0.3 ± 0.02	[7.5]
+ 1 μM Quercetin	0.02 ± 0.01	[0.5]	4 ± 0.05	[100.0]
+ 5 μM Quercetin	0.03 ± 0.01	[0.8]	1 ± 0.01	[25.0]
+ 10 μM Quercetin	0.02 ± 0.01	[0.5]	0.6 ± 0.01	[15.0]
+ 1 μM Rutin	0.03 ± 0.01	[0.8]	6 ± 0.05	[150.0]
+ 5 μM Rutin	0.02 ± 0.01	[0.5]	3 ± 0.01	[75.0]
+ 10 μM Rutin	0.02 ± 0.01	[0.5]	0.7 ± 0.01	[17.5]
+ 1 μM E3G	0.02 ± 0.01	[0.5]	5 ± 0.04	[125.0]
+ 5 μM E3G	0.03 ± 0.01	[0.8]	3 ± 0.02	[75.0]
+ 10 μM E3G	0.02 ± 0.01	[0.5]	1 ± 0.02	[25.0]
+ 1 μM Tamarixetin	0.03 ± 0.01	[0.8]	6 ± 0.03	[150.0]
+ 5 μM Tamarixetin	0.02 ± 0.01	[0.5]	4 ± 0.02	[100.0]
+ 10 μM Tamarixetin	0.02 ± 0.01	[0.5]	2 ± 0.01	[50.0]

**Fig. 6:** Chemosensitizing potential of the selected flavonoids in drug-resistant MCF-7/ADR cell lines. Concentration-dependent curves of doxorubicin with or without flavonoids (1,5 and 10 μM) in parental MCF-7 and MCF-7/ADR cell lines were constructed. The IC_50_ values of MCF-7/ADR cell lines were compared with parental MCF-7 cells. Data denotes the mean ± S.E.M of four experiments, each done in triplicate

**Fig. 7:** Flavonoids downregulate mdr1 expression through wnt/β-catenin signaling pathway

**Table 2:** The concentration of flavonoid necessary for 50% inhibition (IC_50_ values) for cell viability was revealed. Mean ± SEM are from four analytical experiments which were performed in triplicate. bFR: fold-drug resistance was derived by dividing the IC_50_ concentration for doxorubicin of MCF-7 and MCF-7/ADR cells in the absence/presence of theaflavin, quercetin, rutin, epicatechin 3 gallate and tamarixetin by the IC_50_ concentration for doxorubicin of MCF-7 cells

Compound	MCF-7		MCF-7/ADR	
	IC_50_ ± SEM^α^ (μM)	FR^b^	IC_50_ ± SEM^α^ (μΜ)	FR^b^
Doxorubicin	0.32 ± 0.01	[1.0]	8.57 ± 0.23	[26.78]
+ 1 μM Theaflavine	0.32 ± 0.02	[1.0]	5.31 ± 0.04	[16.57]
+ 5 μM Theaflavine	0.29 ± 0.01	[0.9]	3.12 ± 0. 03	[9.75]
+ 10 μM Theaflavine	0.27 ± 0.01	[0.8]	0.8 ± 0.02	[2.5]
+ 1 μM Quercetin	0.31 ± 0.02	[0.9]	5.9 ± 0.05	[18.43]
+ 5 μM Quercetin	0..29 ± 0.02	[0.9]	3.41 ± 0.01	[10.65]
+ 10 μM Quercetin	0.28 ± 0.01	[0.8]	1.1 ± 0.01	[3.43]
+ 1 μM Rutin	0.32 ± 0.03	[1.0]	6.8 ± 0.05	[21.25]
+ 5 μM Rutin	0.30 ± 0.01	[0.9]	4.5 ± 0.01	[14.06]
+ 10 μM Rutin	0.28 ± 0.01	[0.8]	1.6 ± 0.01	[5.0]
+ 1 μM E3G	0.32 ± 0.02	[1.0]	6 ± 0.04	[18.75]
+ 5 μM E3G	0.31 ± 0.01	[0.9]	3.8 ± 0.02	[11.87]
+ 10 μM E3G	0.29 ± 0.02	[0.8]	1 ± 0.02	[3.12]
+ 1 μM Tamarixetin	0.32 ± 0.02	[0.8]	7.3 ± 0.03	[22.81]
+ 5 μM Tamarixetin	0.31 ± 0.02	[0.5]	4.9 ± 0.02	[15.31]
+ 10 μM Tamarixetin	0.30 ± 0.01	[0.5]	2.53 ± 0.01	[7.9]

## Conclusion

Collectively, flavonoids enhanced doxorubicin efficacy through modulating Wnt/β-catenin signaling, downregulating ABCB1 overexpression and augmenting doxorubicin-induced G2/M arrest and apoptosis in multidrug-resistant KBCH^R^8–5 cells. Thus, flavonoids may be considered as an MDR reversal agent after confirming in vivo chemosensitizing potential in preclinical animal models.

## Additional files

Additional file 1: **Figure S1**. A) Pymol outlook of ligand binding domain (LBD) of GSK 3β with quercetin. B) Ligplot image illustrate hydrogen and hydrophobic bonding of GSK 3β with quercetin (ii). A) Pymol outlook of the ligand binding domain (LBD) of GSK 3β with rutin. B) Ligplot image indicates hydrogen bonding and hydrophobic interactions of GSK 3β with rutin (iii). A) Pymol outlook of the ligand binding domain (LBD) of GSK 3β with epicatechin 3 gallate. B) Ligplot view of hydrogen and hydrophobic bonding of GSK 3β with epicatechin 3 gallate. (iv). A) Pymol image show of the ligand binding domain (LBD) of GSK 3β with tamarixetin. B) Ligplot image illustrate hydrogen and hydrophobic interactions of GSK 3β with tamarixetin. **Figure S2.** Wnt, GSK 3β and β-catenin mRNA and protein expression levels in KB3–1 and KBCH^R^8–5 cell lines. Expression levels were normalized with the expression pattern of β-actin levels. Data are given as mean ± SEM of three independent experiments. Data not sharing a similar marking (a, b…) differ significantly at *P* < 0.05 vs. control (DMRT). **Figure S3.** Quantification of protein and RNA are depicted as graph. The densitometry values show means ± SD from three independent immunoblots. The relative density of protein expression levels were normalized to the β-actin protein expression pattern. The mRNA expression pattern was normalized with 18S and the image illustrates quantification of three independent analysis (means ± S.D). Data not showing a similar symbol differ significantly at *p* ≤ 0.05 (DMRT). **Table S1.** Induced-fit docking of flavonoids against GSK 3β. Docking analysis was carried out for 5 flavonoids, which show glide energy, docking score, hydrogen bond interactions. The tested flavonoids exhibit strong inter- and intramolecular interactions with drug-binding pocket of GSK 3β. (DOC 808 kb)

## Abbreviations

ABCB1: ATP-binding cassette sub-family B member 1
APC: Adenomatous polyposis coli
BAX: BCL2-Associated X Protein
BCL-XL: B cell lymphoma-extra large
CDK2: Cyclin-dependent kinase 2
CDKN1A: Cyclin-dependent kinase inhibitor 1A
FZD: Frizzled 1
GSK 3β: Glycogen synthase kinase 3β
LBD: Ligand Binding Domain
LRP: Lipoprotein receptor-related protein
MDR1: Multidrug resistance protein 1
MTT: 3-(4,5-Dimethylthiazol-2-Yl)-2,5-Diphenyltetrazolium Bromide
PBS: Phosphate buffered saline
PDB: Protein Data Bank
P-gp: P-glycoprotein
PI: Propidium iodide
qRT-PCR: Quantitative real-time polymerase chain reaction
RCSB: Research Collaboratory for Structural Bioinformatics
Wnt: Wingless-related integration site
